RETRACTED

# The Effect of Narrative Nursing Intervention on Shame in Elderly Patients with Bladder Cancer after Ileal Bladder Replacement: A Cohort Study

**DOI:** 10.1155/2022/4299919

**Published:** 2022-06-30

**Authors:** Lang Wang, Dan Wu, Shufang Wu, Ya Liu, Xiaoxi Tan, Yun Liu, Ziyuan Wu, Qian Wang, Xiachan He

**Affiliations:** Clinical Nursing Teaching and Research Section, The Second Xiangya Hospital, Central South University, Changsha, Hunan Province, China

## Abstract

**Background:**

The standard treatment for bladder cancer (BC) is transurethral resection (TURBt), intravesical chemotherapy, and regular follow-up cystoscopy after surgery. However, some patients experience relapse or progression. Narrative care refers to a nursing model in which nurses put themselves into the patient's position through communication and listening, thereby alleviating the patient's negative emotions. This study analyzed narrative nursing interventions in elderly patients with BC after vesicoileal replacement.

**Objective:**

To explore the positive stimulating effect of narrative nursing intervention on the sense of shame in elderly patients with bladder cancer (BC) after ileal bladder replacement.

**Methods:**

A total of 60 elderly patients with BC who went through ileal replacement of the bladder from February 2019 to April 2021 in our hospital were enrolled. The patients were divided into the control group and the study group by the arbitrary number table method. The former group received routine care, and the latter group received a narrative nursing intervention model. The nursing satisfaction, stigma score, self-care ability score, SAS score, SDS score, and quality of life score were compared.

**Results:**

First, we compared the nursing satisfaction. In the research group, 23 cases were very satisfied, 6 cases were satisfied, and 1 case was normal, and the satisfaction rate was 100.00%. In the control group, 13 cases were very satisfied, 8 cases were satisfied, 4 cases were general, and 5 cases were dissatisfied, with a satisfaction rate of 83.33%. The nursing satisfaction of the research group was significantly higher compared to that of the control group (*P* < 0.05). Secondly, we compared the stigma scores. The stigma scores of the study group at the time of discharge, 1 month, 3 months, and 6 months after discharge were lower compared to those of the control group (*P* < 0.05). In terms of the scores of self-care ability, the total scores of self-concept, self-care responsibility, self-care knowledge, self-care skills, and self-care ability of the research group were higher compared to those of the control group (*P* < 0.05). With regard to SAS scores, before nursing, there was no significant difference exhibited (*P* > 0.05). After nursing, the patient's SAS score decreased. Compared with the two groups, the SAS scores of the study group at discharge, 1 month, 3 months, and 6 months after discharge were all lower (*P* < 0.05). In terms of SDS score, there was no significant difference before nursing (*P* > 0.05). After nursing, the SDS scores of patients decreased. Compared between the two groups, the SDS scores of the study group at the time of discharge, 1 month, 3 months, and 6 months after discharge were lower (*P* < 0.05). Finally, we compared the life quality scores. Before nursing, there was no significant difference exhibited (*P* > 0.05). After nursing, the scores of life quality of patients improved. Compared with the two groups, the physical function, psychological function, social function, and healthy self-cognition scores of the research group were all lower compared to those of the control group (*P* < 0.05).

RETRACTED

**Conclusion:**

Narrative nursing can reduce anxiety and depression in elderly patients with BC after ileal replacement of the bladder, enhance the quality of life, reduce the patient's stigma, and play a positive motivating role. This nursing model is worthy of promotion in clinic.

## 1. Introduction

Bladder cancer (BC) is a common urogenital malignancy [1–4]. There is no effective treatments for BC currently. The standard treatment for BC is transurethral resection (TURBt), intravesical chemotherapy, and regular review of cystoscopy after surgery. However, some patients (about 50%-80%) will experience the recurrence or progression [2]. Muscle-invasive BC (MIBC) are more likely to have distant metastases and worse outcomes. At present, the primary therapy for MIBC is still radical cystectomy and urinary diversion [3]. The main side effect of urinary diversion surgery is the inability of most patients to voluntarily control their urine after surgery. Therefore, some patients choose TURBT because they cannot accept the disadvantage of not being able to control their urine after surgery [4]. At present, there are mainly the following types of urinary diversion: ileal bladder, ureterostomy, percutaneous urinary diversion, and urinary control by the anus [5]. Ileal bladder surgery is seen as a classic simple, safe, and effective method of choice for uncontrollable urinary diversion, and it is also one of the most commonly used methods of urinary diversion. Ureter cutaneous ostomy is another simple and safe operation, suitable for patients with short life expectancy, distant metastasis, palliative cystectomy, bowel disease unable to use bowel for urinary diversion, or systemic conditions who cannot tolerate surgery. In recent years, clinical medical staff have gradually started to realize that the evaluation of the therapeutic effectiveness of cancer patients is not only to prolong the survival time but also to satisfy the patients' needs such as the health-related life quality. Although ileal bladder surgery is an effective method to save the patient's life and relieve the patient's symptoms, the psychological and physical changes in the patient cause great mental stress and negative emotions, resulting in inconvenience to the patient's life [6].

RETRACTED

Humanistic care for oncology patients is gaining popularity, so narrative care is gradually implemented in clinics [7]. It mainly refers to the nursing model in which nursing staff bring themselves into the patient's position through communication and listening, understand the patient's actual problems, assist in resolving the patient's problems, and thus alleviate negative moods [8, 9]. Narrative care varies from person to person and can profoundly address the problems of patients with various diseases and cultural backgrounds, improving the effectiveness of psychotherapy. However, it is still in its infancy. In this study, the narrative nursing intervention on elderly patients with BC after ileal replacement of the bladder was analyzed.

## 2. Patients and Methods

### 2.1. Patient Information

A total of 60 elderly patients with BC who went through ileal replacement of the bladder from February 2019 to April 2021 in our hospital were enrolled. The patients were divided into the control group and the study group by the arbitrary number table method. The former group received routine care, and the latter group received a narrative nursing intervention model. In the control group, the age ranged from 64 to 85 years old, with an average age of70.58 ± 4.33years old, including 18 males and 12 females. In the research group, the age ranged from 44 to 76 years old, with an average of 65.96 ± 3.58 years old, including 16 males and 14 females. The general data of patients were not statistically significant. This study was permitted by the medical ethics committee of our hospital, and all patients provided informed consent.

The selection criteria are as follows: (1) age ≥ 60 years old; (2) no cognitive, language, and intellectual dysfunction, with basic reading and writing skills; (3) inpatients in the rehabilitation period after radical cystectomy and ileocystostomy for BC; and (4) able to complete this questionnaire independently.

The exclusion criteria are as follows: (1) no reading ability; (2) patients with more than second hospitalization after ileocystostomy; (3) questionnaire answers are obviously not considered to answer (the answers are regular or the answer options are the same); and (4) patients with a history of mental illness.

RETRACTED

### 2.2. Treatment Methods

The control group received routine nursing intervention in the department. On the day of admission, patients in the control group received the department's disease guidebook, admission assessment, and health education.

On the basis of the control group, the research group implemented narrative nursing intervention. The specific measures are as follows: (1) set up a narrative nursing research group. The research team consists of 2 psychologists, both of whom are national second-level psychological consultants, who are responsible for training the members of the narrative nursing team and solving the professional problems encountered in the narrative process; one head nurse is responsible for the overall planning, organizing the study and assessment of team members, coordinating the work schedule of nurses in the group, supervising the work and quality control during the group research process, and solving problems in the actual operation process; the researcher himself engaged in clinical nursing. There are 4 nurses in charge who have worked for more than 5 years and have passed the psychological counselor exam, serving as narrative nurses, responsible for implementing one-to-one narrative nursing interventions for patients from admission to follow-up after discharge. The psychology team of our school also provided strong theoretical support and technical guidance for this research; (2) training methods: (1) before the intervention, set up a research group Ding Talk group, and independently learn Li Chun's voice version of “Hundred Days of Narrative Nursing Micro-Lessons” through the WeChat platform and *Communication Technology* book; psychologists take turns to train narrative nursing online every Monday and Thursday, about 40 minutes each time, for a total of 12 weeks. The training content includes the meaning of narrative nursing, core techniques of narrative nursing, including externalization, deconstruction, rewriting, external witnesses, and treatment documents, to learn the relevant knowledge of narrative nursing, so that they can fully understand the concept, meaning, intervention methods, and communication skills of narrative nursing, clinical application, etc., to cultivate nurses' narrative ability and standardized communication ability; (2) invite the professor of psychology department of our hospital to explain “Introduction to Narrative Therapy” for about 90 minutes. Contents include treatment methods of postmodern psychology, postmodern psychological theory, social construction theory, and history of narrative therapy; invite national second-level psychological counselors to teach the difference between narrative therapy and traditional psychotherapy, the counseling structure of narrative therapy, and narrative therapy with clinical application; the time is about 90 min. This video is synchronized to the research group; (3) practice assessment: while the team members continue to deepen the knowledge of narrative nursing, psychologists set up cases, conduct scenario simulations, give guidance on the problems existing in the process of narrative nursing for nurses, and conduct assessment and evaluation, with a score of more than 90 points to participate in the research. The nurse writes a reflection diary and shares it with the Ding Talk group.

RETRACTED

*Narrative nursing*: follow the narrative nursing procedures to focus, understand, reflect, and respond, and comprehensively use the five core technologies of externalization, deconstruction, rewriting, external witnesses, and treatment documents. Under the premise, choose an appropriate time in the location of classroom, single ward, or conference room; and avoid patients' meal and rest time; conduct one-to-one, face-to-face communication to ensure a quiet and confidential environment during the interview 3 times a week, 30-45 min each time, for a total of 5-6 times during hospitalization. To reduce bias, narrative nursing was performed on the same subjects by the same nurse in the research team as the narrative nurse. (1) Concern stage: it is the primary work content of narrative nursing work. Nurses collect data to fully understand their family background, educational experience, religious belief, hobbies, personality characteristics, work status, and economic income. Choose the right time; communicate with the patient in advance; establish a trusting relationship; guide the patient to say the things that make them feel most painful, troubled, anxious, and depressed; and express their true feelings. For example, we could start with: “I don't think you're in a good mood, is there something you're not happy about? Can you talk to me?” “You're not very talkative, is this always the case or is there something you're having trouble with? It might be more comfortable to say it.” “Is there anything you want to talk to me about?” At this stage, the following points should be paid attention to: (1) establish an attitude of reverence for life, put yourself in a position of equal treatment with patients, do not comment on the right or wrong of the problems raised by patients, and aim to guide patients to express their true feelings. Talk about negative emotions, and let patients know that they are willing to take the time to listen and build trusting relationships; (2) nurses have keen observation skills; they not only pay attention to the progress of the patient's physical disease but also carefully observe the patient's expressions, demeanor, movements, and other nonverbal behaviors; (3) use empathic listening skills at this stage; play the role of nonverbal behavior; maintain proper eye contact with the intervention object throughout the process; allow the patient to cry; listen patiently, without interruption or correction; and encourage them to fully narrate a certain situation as much as possible. One thing, express the most real feelings and thoughts in the heart, and completely vent the emotions. (2) Comprehension stage: the narratives carried by the patients are usually fragmented, messy, and illogical. To correctly understand the patients' narratives, nurses need to use specific narrative nursing techniques in addition to having an attitude of empathy, including (1) deconstructing the narrative elements of the patient's story, such as time frame, event context, and occurrence process; (2) pay attention to the social and cultural factors contained in the background of the story; (3) dig deeply and imaginatively interpret the facilitating or hindering factors in the narrative, and identify the deep meaning hidden in the patient's narrative; (4) sympathy and understanding of the painful experiences and experiences the patient narrates. For example, when the subject stops talking in the middle of the conversation, you can say something like: “I understand your thoughts very well, can you talk a little more? What was your family like when that happened?” “How were you? See how that event changed your life?”; (3) reflection stage: before responding to the patient's narrative, nurses reflect on their own cognition, understanding, and handling of the patient's disease narrative, and summarize their own problems, including (1) thinking about the stable value orientation, interests, prejudices, emotional attitudes that have been formed by oneself, and the influence of these factors in the process of paying attention to and understanding the patient's narrative; (2) examining their premade assumptions and judgments about the patient's narrative; explaining whether there is any deviation; (3) eliminate inappropriate emotions and habits that affect oneself to make correct thinking and nursing countermeasures. Through reflection, narrative nurses can recognize their prejudice against the research object and should enter the research object's story with an inclusive and understanding mentality, understand the research object, and show respect for it. (4) Response stage: it is the core of narrative nursing intervention. Narrative nurses can respond to the research object in two ways. One is timely response; that is, they respond to the emotions expressed by the research object during the narrative process, by soothing touch, smiling, nodding, etc.; the other is delayed response; that is, the narrative nurse designs a specific and complete response plan after in-depth analysis of the narrative content of the research subject; the methods are as follows: (1) externalization problem. Help the research subject separate himself from the problem, make the problem concrete, let him know that the problem and himself are two different individuals, focus on the disease or problem, fully clarify the state of the disease or problem, and increase the number of research subjects; the sense of control over the problem is the most characteristic treatment method and technique of narrative therapy. You can ask the research subjects to choose a name that is close to their own experience according to their current state, such as “trouble,” “big rock,” “heavy,” and “loneliness”; “When did this “big rock“ in the heart appear?” “What does that ‘trouble' look like? Can you describe it?” “How long has your ‘loneliness' been around?” “The separation of people and problems is achieved through naming; (2) deconstructing the problem. Explore the history, impact, and outcomes of the problem with the research subject; explore the sociocultural context behind the subject's problem or behavior; and enable it to see how the problem is constructed and how it is affected by unnoticed social values and ideas. Influenced by hypotheses, it helps the research subjects to jump out of the inherent thinking influenced by the mainstream culture and obtain the possibility of looking at problems from different perspectives. Ask the research subjects why they have a certain idea, during which they will touch people's self-identity. Through the answers of the research subjects, the deep-level social and cultural factors behind the cognition and thinking will be excavated. For example, “What has changed in this big rock? When is it strong? When is it weak?” “How did loneliness come about? How did you get along with it after coming here?” “Why do you think so? Why do you think are you such a person?” “Have you encountered a similar situation before? How did you solve it then?”; (3) rewrite the event. Guide the research subjects to find positive events from painful experiences as exceptional events, and give positive praise and positive comments to the positive qualities of the research subjects in exceptional events, such as optimism, bravery, seriousness, and ability. Encourage and inspire them to explore their own potential and enhance their determination to solve problems. For example, by questioning the subject, we learned that he won the first place in the district when he was at school, completed a huge order after work, and was rewarded by the leaders of the company. Through careful observation and trial three years ago, he properly handled the contract dispute with the company, so that the company avoided economic losses. These are a few exceptions. The narrative nurse can say something like “You can get the first place in the district when you go to school, and you can complete tasks that only a few people can complete after work. What kind of quality do you have?” The narrative nurse guides the research subjects to make a positive evaluation of themselves by asking questions after the research subjects say the exceptional events. This is a branch story after the exceptional events are connected. Then, give guidance: “If you have such excellent qualities (specify your excellent qualities), what will you do when faced with the current problem?” Defer the research object's positive evaluation of yourself to the existing problem, guide the research subjects to make decisions for themselves, and formulate an implementation plan, which is to replace the main story with a side story, and complete the process of rewriting; (4) external witnesses. During the implementation of narrative care, with the consent of the research subjects, family members or other important people of the research subjects can be invited to watch the narrative process and give psychological support and encouragement to the research subjects, such as: “Who do you admire most? He will give you what power?” “Who would be proud of your achievements?” But external witnesses vary, and not every research subject needs an external witness; (5) treatment files. Narrative nurses use a tool to reinforce the subject's beliefs for therapeutic purposes. There are various forms of treatment documents. According to the character of the research subjects, brochures, certificates of merit, audio-visual materials, or WeChat Moments can be given. For example, for the research subjects who are troubled by insomnia, with the help of the narrative nurses, if they sleep well that night, they can post a small smiley face on the record book; if they sleep well for 1 week, they can post a big smiley face to encourage research target and strengthen their confidence in getting out of the predicament and overcoming the existing difficulties. (5) Postdischarge intervention: after the patient was discharged from the hospital, in addition to the routine discharge guidance, the same nurse in the research team had a telephone conversation with the patient, 2 times a week, about 30 minutes each time, for a total of 6 times. The contents include (1) general condition inquiry: inquire about the patient's recent physical condition, sleep quality, discomfort symptoms, or other adverse events in a concerned manner; (2) supervision of rehabilitation goals: Ask the patient about the implementation of individualized rehabilitation goals. If the implementation is poor, discuss with the patient the problems that hinder the implementation of the goal, help the patient find a solution, and provide care and support; if the implementation is good, praise the patient appropriately, and encourage patients to make persistent efforts; (3) psychological assessment: through (1, 2) the emotional state of the patient in the process to evaluate the patient's psychological state; if the patient shows negativity or anxiety, then through patient listening and appropriate inquiry, guide the patient to say the source of negativity or anxiety, respond to each other's feelings with an understanding and receptive attitude, and apply narrative nursing technology to carry out individual psychological counseling; (4) if the phone number of an individual patient cannot be reached, the nurse will mark it and conduct a supplementary conversation in time. It should be noted that in the process of implementing narrative nursing, various stages can be interspersed and overlapped with each other, and they are not completely independent. It is necessary to tap the potential of the patient and provide the basis for narrative nursing according to the actual situation of the patient.

RETRACTED

### 2.3. Observation Indicator

#### 2.3.1. Satisfaction

After reviewing the literature and discussing with experts, design patient follow-up satisfaction, a total of 10 items, and record patients' satisfaction with follow-up management mode, health education, medical service, and appointment registration process [10]. It is assigned into four dimensions: very satisfied, satisfied, general, and dissatisfied. Satisfaction rate = very satisfied rate + satisfaction rate + general rate.

#### 2.3.2. Disgrace Scale

The Chinese version of Stigma Scale for Chronic Illness (SSCI) [11]. It was translated into Chinese by the National Institute of Neurology and Stroke (NINDS) in 2016, and the Chinese version of the scale was used with the consent of the original scale development agency. The scale includes two parts: internal stigma and external stigma, 13 items for internal stigma and 11 items for external stigma. All entries are forward entries. The five options of the scale are never, rarely, sometimes, often, and always, with 1-5 points, respectively, with a full score of 24-120 points. The higher the score, the higher the level of stigma. The Cronbach alpha coefficient of the scale is 0.97, and the reliability and validity are good, and the item test theory test has a good fitting model.

RETRACTED

#### 2.3.3. Urostomy Self-Care Scale

The Kristensen Urostomy Self-Care Scale [12] (Introduction the Urostomy Self-Care Scale) is a standardized tool, compiled by Kristensen et al. in self-care ability. The item measures the patient's self-care willingness and measures the patient's self-care skills. Each entry is assigned into 4 levels, scored from 0 to 3. A score of 0 indicates that the patient is completely dependent on the nurse, and the nurse completes various operations; 1 score indicates that patients participate in nursing skills but need the help of nurses; 2 points indicate that patients need to complete nursing skills under the oral guidance of nurses; 3 points indicate that patients can complete nursing skills independently. The total score was 21, and the higher the score, the higher the self-care level of the patients.

#### 2.3.4. Self-Rating Anxiety Scale

Self-rated anxiety scale [13] (SAS), was compiled by Zung in 1971, including 20 items; each item reflects an anxiety-related symptom, using a 4-point scoring method; the 5th, 9th, 13th, 17th, and 19th items are reverse scores; and the final 20 items' summary scores are multiplied by 1.25 and rounded to the nearest integer, which is the SAS standard score. Higher standard scores indicate more severe anxiety symptoms. The scoring standard is as follows: <50 points, no anxiety; 50-59 points, mild anxiety; 60-69 points, moderate anxiety; and >69 points, severe anxiety. Cronbach's alpha for this questionnaire was 0.91.

#### 2.3.5. Self-Rating Depression Scale

Self-rating depression scale [14] (SDS) was developed by Zung in 1965; a total of 20 items were included, using 4-grade scoring method, in which items 2, 5, 6, 11, 12, 14, 16, 17, 18, and 20 were reverse scores, and finally, each item was multiplied by 1.25 to get the standard total score. The higher the standard total score, the more severe the depression. The SDS scoring standard is as follows: <53 means no depression; 53-62 means mild depression; 63-72 points into moderate depression; and >72 points into severe depression. The Cronbach *α* for this questionnaire was 0.73.

#### 2.3.6. Quality of Life Scale

The scale of life quality [15] consists of four subscales, including physical, psychological, social, and health self-awareness, with a total of 29 items. The Cronbach *α* coefficient of the scale is 0.79-0.91. The scale was scored by 1-5 grades. The lower the score, the higher the satisfaction.

RETRACTED

### 2.4. Statistical Analysis

In this study, Excel 2010 software was employed to establish a database, and after entering the SPSS25.0 database, SPSS25.0 software was adopted for data analysis. (1) Statistical description part: Kolmogorov-Smirnov test was employed for normality test. Measurement data in general demographic data and clinical data that conformed to normal distribution were described by mean ± standard deviation ($\bar{x}\pm \text{s}$), which did not conform to normal distribution. The measurement data are described by quartiles; the count data are expressed by frequency and percentage. (2) Statistical inference: when comparing the baseline data of the two groups of subjects, the measurement data that conformed to normal distribution and equal variance were compared using two independent samples *t* test, and the measurement data that did not conform to the normal distribution adopted the Wilcoxon rank sum test. The statistic is *Z*; enumeration data were analyzed by the chi-square test or exact probability method. Two-sided test was adopted, and the significance level of statistical test was *P* < 0.05, indicating that there was a significant statistical difference exhibited. Repeated-measures analysis of variance was employed to analyze the scores of outcome indicators at each time point before and after intervention of subjects.

## 3. Results

### 3.1. Comparison of Nursing Satisfaction

First, we compared the nursing satisfaction. In the study group, 23 cases were very satisfied, 6 cases were satisfied, and 1 case was normal, and the satisfaction rate was 100%. In the control group, 13 cases were very satisfied, 8 cases were satisfied, 4 cases were general, and 5 cases were dissatisfied, with a satisfaction rate of 83.33%; Comparing the two groups, the nursing satisfaction of the research group was higher than that of the control group, and the difference was statistically significant (*P* < 0.05). All data results are indicated in Figure 1.

#### 3.1.1. Comparison of the Stigma Score between Two Groups

Secondly, we compared the stigma score. The stigma score of the study group on the day of discharge, 1 month, 3 months, and 6 months after discharge was lower compared to that of the control group, and the difference was statistically significant (*P* < 0.05). All the data results are indicated in Figure 2.

### 3.2. Comparison of Self-Care Ability Score

Thirdly, we compared the scores of self-care ability. The total scores of self-concept, self-care responsibility, self-care knowledge, self-care skills, and self-care ability of the study group were higher compared to those of the control group, and the difference was statistically significant (*P* < 0.05). All data results are indicated in Table 1.

RETRACTED

### 3.3. Comparison of SAS Score

Then, we compared the SAS scores. Before nursing, there was no significant difference exhibited (*P* > 0.05). After nursing, the SAS scores of patients decreased. Compared between the groups, the SAS scores of the study group at the time of discharge, 1 month, 3 months, and 6 months after discharge were lower, and the difference was statistically significant (*P* < 0.05). All data results are indicated in Table 2.

### 3.4. Comparison of SDS Score

Next, we compared the SDS scores. Before nursing, there was no significant difference exhibited (*P* > 0.05). After nursing, the SDS scores of patients decreased. Compared between the two groups, the SDS scores of the study group at the time of discharge, 1 month, 3 months, and 6 months after discharge were lower, and the difference was statistically significant (*P* < 0.05). All data results are indicated in Table 3.

### 3.5. Comparison of Quality of Life Score

Finally, we compared the life quality scores. Before nursing, there was no significant difference exhibited (*P* > 0.05). After nursing, the life quality scores of patients decreased. Compared with the two groups, the physical function, psychological function, social function, and healthy self-cognition scores of the research group were all lower, and the difference was statistically significant (*P* < 0.05). All data results are indicated in Table 4.

## 4. Discussion

Bladder cancer is a common clinical disease and one of the common malignant tumors in the urinary system [16]. In my country, the incidence of BC in men ranks 7th among systemic malignant tumors, and that in women ranks after the 10th place [17]. The Cancer Genome Atlas (TCGA) project has enhanced our understanding of BC [18]. The treatment of BC is mainly surgery, and the appropriate surgical method is enrolled according to the clinical stage, pathology of the tumor, and the general condition of the patient [19]. Postoperative abdominal stoma is required, and a urine collection bag is worn for life [20]. Although elderly BC patients undergoing ileal bladder replacement surgery can achieve certain therapeutic effects, if new targeted nursing interventions can be given, they can effectively enhance the negative emotions of patients and have a positive impact on patients' lives [21].

Narrative nursing, as a new approach to clinical psychological nursing that is highly compatible with humanistic attributes, means that medical workers can provide respectful, vibrant, and empathetic medical care by recognizing, absorbing, responding to patients' dilemmas, nursing, helping patients rebuild a new life style, and then discovering the points of personalized medical care and implementing interventions for patients [22]. It is helpful for patients to express their concerns, relieve pain in their hearts, and form a positive attitude to face the disease, and the treatment effect is optimistic, which is beneficial to the prognosis of the disease [23]. Influenced by the trend of postmodernism, Australian scholars Michael White and David Epston first proposed narrative therapy in 1980 [24], advocating that the problem lies in the problem itself, rather than the person, emphasizing personal concepts and emphasizing the interpretation of inner emotions, values, and meanings, so as to provide psychological benefits. Since the mid-1980s, the concept of narrative therapy has been gradually promoted from Australia and other places to Europe and Asia and other countries, and from the initial family therapy, it has been gradually applied to AIDS group therapy [25], community culture, schools, hospitals, and other fields to help individual or groups address psychological distress or barriers [26]. At the end of the 20th century, narrative therapy began to be gradually applied in the field of nursing. Scholars such as Fitzpatrick and Ankeet put forward the concept of narrative nursing combined with the characteristics of nursing profession and defined narrative nursing as nurses with narrative ability [27, 28]. Humane and effective nursing practice means nurses understand and respond to patients' suffering and plight, experience and gain insight into patients' feelings and needs, and provide respectful, vital, and empathetic care. At present, the definition of narrative nursing has not been uniformly defined. Wang et al. combined the viewpoints of scholars to propose that narrative nursing refers to a kind of witnessing, absorbing, and a nursing practice model that understands, experiences, and responds to the suffering of patients, which can help patients to reconstruct the meaning of life and disease stories and to discover nursing points [29]. In narrative nursing, the overall nursing concept of “patient-centered” is reflected, and stories are used to inspire patients to express their emotions, which helps patients express their concerns, relieve inner pain, and ultimately benefit the prognosis of the disease [30].

RETRACTED

Narratives are a way for patients to tell the illnesses and traumatic events they have experienced, revealing not only physical pain but also psychological distress, such as fear, anxiety, self-acceptance disorders, and interpersonal changes [31]. Most patients have a tendency to confide, and they sometimes confide details of their disease stories to relatives, friends, medical staff, and even strangers. The patient narrative is not a simple statement of life events but is full of their painful, dazed, and even open-minded emotional experience. Guiding patients' narratives and using the cathartic effect of patients' narratives to relieve inner pain and ultimately benefit the prognosis of the disease are two of the key points of clinical intervention using narrative nursing [32]. At the nursing and health education level, narrative is an emerging and persuasive method that is often used to use the stories of others or specific behavioral groups to inspire behavioral or thinking changes in target groups. Narrative nursing can become an effective health education method because of the characteristics of the narrative itself, that is, communication, homogeneity, behavior orientation, and reality. Stories are the practical carriers of narrative intervention methods, and stories often have the power to face people's hearts and can deeply convey the goals and concepts of health education. Narrative is the nexus of the nurse-patient relationship. In clinical work, nurses have more time to spend with patients than doctors and have the opportunity to understand patients' stories. Narrative nursing requires nurses to actively listen to and appropriately respond to patients' stories. When patients feel understood, they will have a deep sense of satisfaction and thus, it promotes the establishment of a nurse-patient emotional alliance. The nurse-patient alliance based on emotional identity and treatment cooperation is the most stable and reliable relationship between nurses and patients.

In summary, narrative nursing can reduce anxiety and depression after ileal bladder replacement in elderly BC patients, improve quality of life, reduce patients' shame, and play a positive motivating role. This nursing model is worthy of clinical promotion.

## Figures and Tables

**Figure 1:** Comparison of nursing satisfaction between two groups. Comparing the two groups, the nursing satisfaction of the research group was higher than that of the control group, and the difference was statistically significant (*P* < 0.05).

**Figure 2:** Comparison of the stigma score between two groups. The stigma score of the study group on the day of discharge, 1 month, 3 months, and 6 months after discharge was lower compared to that of the control group, and the difference was statistically significant (*P* < 0.05).

**Table 1:** Comparison of self-care ability scores of patients ($\bar{x}\pm \text{s}$, points).

Group	*N*	Self-concept	Sense of self-care responsibility	Self-care knowledge	Self-care skills	Total score
C group	30	20.19 ± 1.23	12.58 ± 3.44	28.19 ± 1.21	24.59 ± 1.21	94.19 ± 2.45
R group	30	25.39 ± 2.21	19.39 ± 2.42	33.19 ± 4.42	28.15 ± 3.31	106.38 ± 2.43
*t*		11.260	8.868	5.976	5.532	19.348
*P*		<0.01	<0.01	<0.01	<0.01	<0.01

RETRACTED

**Table 2:** Comparison of SAS scores between the two groups of patients ($\bar{x}\pm \text{s}$, points).

Group	*N*	Before nursing	On discharge	1 month after discharge	3 months after discharge	6 months after discharge
C group	30	65.91 ± 3.91	56.95 ± 5.22	50.81 ± 2.21	46.39 ± 1.35	41.28 ± 1.22
R group	30	65.95 ± 3.64	52.92 ± 3.31	45.19 ± 1.33	40.86 ± 3.45	34.58 ± 2.12
*t*		0.041	3.571	11.934	8.175	15.003
*P*		>0.05	<0.01	<0.01	<0.01	<0.01

**Table 3:** Comparison of SDS scores between the two groups of patients ($\bar{x}\pm \text{s}$, points).

Group	*N*	Before nursing	On discharge	1 month after discharge	3 months after discharge	6 months after discharge
C group	30	67.39 ± 3.12	62.39 ± 2.24	59.91 ± 1.33	54.93 ± 3.31	45.96 ± 2.14
R group	30	67.94 ± 3.31	60.19 ± 1.34	54.91 ± 3.52	49.19 ± 4.23	40.69 ± 3.31
*t*		0.662	4.616	7.277	5.853	7.323
*P*		>0.05	<0.01	<0.01	<0.01	<0.01

**Table 4:** Comparison of life quality scores between the two groups of patients before treatment ($\bar{x}\pm \text{s}$, points).

Group	*N*	Physiological function		Mental function		Social function		Healthy self-awareness	
		Before nursing	After nursing	Before nursing	After nursing	Before nursing	After nursing	Before nursing	After nursing
C group	30	15.84 ± 4.91	13.86 ± 2.95^a^	16.94 ± 3.91	14.85 ± 4.86^a^	18.82 ± 3.95	16.37 ± 2.81^a^	15.98 ± 3.91	13.86 ± 1.85^a^
R group	30	15.96 ± 4.52	11.84 ± 2.91^b^	16.95 ± 3.86	12.81 ± 1.85^b^	18.84 ± 3.55	12.84 ± 3.81^b^	15.87 ± 3.66	10.83 ± 2.91^b^
*t*		0.098	2.670	0.009	2.148	0.020	4.084	0.112	4.812
*P*		0.921	0.009	0.992	0.035	0.983	<0.01	0.910	<0.01

Note: comparison before and after nursing in the control group, ^a^*P* < 0.05; comparison before and after nursing in the study group, ^b^*P* < 0.05.

## Data Availability

No data were used to support this study.
